The article "The Use of System Dynamics Methodology in Building a COVID-19 Confirmed Case Model" was published in 2020. Journal: Comput Math Methods Med.

# The Use of System Dynamics Methodology in Building a COVID-19 Confirmed Case Model

**DOI:** 10.1155/2020/9328414

**Published:** 2020-11-07

**Authors:** Mohd Izhan Mohd Yusoff

**Affiliations:** Telekom Research & Development Sdn Bhd, TM Innovation Centre, Lingkaran Teknokrat Timur, 63000 Cyberjaya, Selangor Darul Ehsan, Malaysia

## Abstract

Researchers used a hybrid model (a combination of health resource demand model and disease transmission model), Bayesian model, and susceptible-exposed-infectious-removed (SEIR) model to predict health service utilization and deaths and mixed-effect nonlinear regression. Further, they used the mixture model to predict the number of confirmed cases and deaths or to predict when the curve would flatten. In this article, we show, through scenarios developed using system dynamics methodology, besides close to real-world results, the detrimental effects of ignoring social distancing guidelines (in terms of the number of people infected, which decreased as the percentage of noncompliance decreased).

## 1. Introduction

The Institute for Health Metrics and Evaluation (IHME) used a hybrid model that combines the estimated hospital resource demand with a disease transmission model to make a forecast of the spread of the disease in the US. This new model captures the impact of changes in social distancing mandates, changes in mobility, and the impact of testing and contact tracing. It enables predicting resurgence if and when more social distancing mandates are relaxed. The model facilitates regular updating as new data of cases, hospitalizations, deaths, testing, and mobility are publicized. It can also be used to identify what may be the trajectory to progressively relax social distancing and, at the same time, limit the risk of large-scale resurgence [1]. Murray et al. [2] determined the extent and timing of deaths and excess demand for hospital services due to COVID-19 in the US and presented the first set of estimates of predicted health service utilization and deaths due to COVID-19, day by day, for the next four months for each state in the US. Using the daily data of confirmed COVID-19 deaths from the WHO websites and local and national governments, data on hospital capacity and utilization for US states, and observed COVID-19 utilization data from select locations, they discovered that even with social distancing measures enacted and sustained, the peak demand for hospital services due to the COVID-19 pandemic is likely to exceed the capacity substantially. Supported by mobile phone data, Murray et al. [3] developed a mixed-effect nonlinear regression framework to estimate the trajectory of the cumulative and daily death rate as a function of the implementation of social distancing measures. An extended mixture model was used to capture asymmetric daily death patterns. These estimates can help inform the development and implementation of strategies to mitigate the load on health system resources, including reducing non-COVID-19 demand for services and temporarily increasing the capacity of the system. They predicted the estimated excess demand on hospital systems within three weeks of implementing social distancing measures in all locations that had not implemented the measures already. They further made similar estimates in case these measures were implemented throughout the epidemic. They emphasized the importance of implementing, enforcing, and maintaining these measures to mitigate hospital system overload and prevent deaths. Using data derived from mobile phone GPS traces, Woody et al. [4] proposed a Bayesian model to project first-wave COVID-19 deaths in all 50 US states and to estimate how social distancing behaviour was causing the “flattening of the curve” in each state. The model outperformed the widely used IHME model. The dynamic SEIR model created by Yang et al. [5] was effective in predicting the COVID-19 epidemic peaks and sizes, and the implementation of control measures on January 23, 2020, in China, which managed to curb the size of the COVID-19 epidemic. Marchant et al. [6] evaluated the IHME model and found that its predictions of the daily number of deaths have been highly inaccurate, especially when predicting the number of next day deaths.

This paper (divided into Methodology, Program, Results, and Conclusion) reports a system dynamics methodology capable of showing the number of people involved in the infections (for example, person “A” infects persons “B,” “C,” and “D”; person “C” in turn infects persons “F,” “G,” “H,” and “I”; and the number of people involved in the infections equals to eight), in a given population and observation period, when changes are made to the percentage of violators (or those who did not practice social distancing) and rate of infection.

## 2. Methodology

System dynamics methodology is defined as a methodology for understanding how things change over time. It focuses on the feedback behaviour of variables within the system's closed loop and deals with how the internal feedback loops within the structure of a system create behaviour. The strength of system dynamics methodology lies in the way it analyses the impact of information feedback on the decision making in a complex system.

Stock, represented by population and COVID-19 confirmed cases in Figure 1, is an element that accumulates and depletes over time. Flow, represented by the rate of infection, is the rate of change in the stock. Link defines a dependency between elements of the stock and flow diagram, and auxiliary, represented by parameters, is used to define some intermediate concepts. Positive feedback loops enhance or amplify changes, which tend to move a system away from its equilibrium state and make it more unstable. Negative feedback loops dampen or buffer changes, which tend to hold a system in a state of relative equilibrium, making it more stable [7]. The (COVID-19 confirmed cases) model (developed using system dynamics methodology as shown in Figure 1) is translated or converted into a program; details are given in the next section.

The stock (typical) behaviour of the system dynamics methodology is exemplified below:

Auxiliary_1, Rate_1, and Level_1 (representing stock) of model “A” in Figure 2 are fixed at (constant value) 10, auxiliary per day, and (initial value) 0, respectively.

Figure 3 shows the results produced by Level_1 when model “A” is executed. Level_1 behaviour can be explained via the following mathematical formula: Level_1_ = (Auxiliary_1_)*t*, *t* = 1, 2, 3, ⋯.

## 3. Program

The program, that is called “covid19curve” and developed using Java programming language, performs the following steps (note that, we relied heavily on assumptions or best guesses because of unavailability of or limited access to real data):

A person is randomly selected to be infected by the virus (representing the scenario or condition where he or she is infected by the virus from the outside population; for example, the person is infected by the virus at a religious gathering held outside the population or community), and the person becomes the source of infection for others (especially those who are “free” from infection and standing less than 6 feet, or 2 meters, away, in other words, not practicing social distancing). The virus is transmitted from person to person when one person comes into contact with an infected person, such as by a handshake or secretions, for example, droplets expelled in a cough or sneeze. It can also be transmitted if one touches the things the infected person has touched and then touches their mouth, nose, or eyes [8]. The said person is labelled as “Source,” and the infected by the “Source” are labelled as “Sink.” The people labelled “Sink” can in turn be labelled as “Source” if they infect others (who are labelled “Sink”). Labels “Source” and “Sink” are used (or introduced) for easy “contact-tracing” exercise (a special or unique feature that is added to the system dynamics methodology's stock labelled “COVID-19 confirmed cases” in Figure 1 and its typical behaviour can be found in Figures 2 and 3). This is similar to the real world where, before the introduction of Malaysia's movement control order (MCO) or Singapore's circuit breaker, or in some cases, people unaware of having been infected (or having mistaken the virus for common or seasonal flu) unwittingly infected others.

The above steps in the program are repeated fifty (50) times for each of the following scenarios. The population and observation period are fixed, respectively, at 1000 and 5 days (the population is labelled as 1, 2, 3,…, 1000). The results from the program could be treated as clusters, for example, a religious gathering or a wedding ceremony. If the number of persons infected is one (1), we are assuming that the person is infected by the virus from outside the population (as mentioned in the previous paragraph). The following scenarios could represent conditions before (i.e., Scenario 1) and during the enforcement of MCO (i.e., Scenario 3) and in the reverse case, that is, after MCO is lifted or relaxed.

Malaysia's MCO was first introduced on 18 March and lasted till 14 April; it was then extended till 28 April and extended again till 12 May 2020. Conditional MCO (CMCO), under which more businesses were allowed to open with strict guidelines or Standard Operating Procedure (SOP), was introduced on 4 May and lasted till 12 May, and it was extended further till 9 June 2020 [9, 10]. Although Enhanced MCO (EMCO) with stricter orders was enforced in several areas in Malaysia (which include blocking the roads with barbed wire), it will not be included in this study. Scenario 2 could represent conditions during the enforcement of CMCO (and before the enforcement of MCO).

*Scenario 1*: approximately 80% of the population did not follow or practice social distancing (maintaining 6-feet, or 2-meter, distance between persons), and the rate of infection follows a statistical distribution, normal (7, 1) [11]. Rate of infection, normal (*μ*, *σ*^2^), is derived from observation period and the percentage of population that did not practice social distancing.

*Scenario 2*: approximately 50% of the population did not follow or practice social distancing (staying 6 feet, or 2 meters, apart from others), and the rate of infection follows statistical distribution, normal (3, 1).

*Scenario 3*: approximately 10% of the population did not follow or practice social distancing (6 feet, or 2 meters, apart), and the rate of infection follows statistical distribution, normal (0, 1).

Box plot [12] (Figure 4) is used to display the results from all scenarios, focusing on the number of people involved in the infections that fulfils the following intervals: between lower hinge and median (H-M), between median and upper hinge (M-H), between lower inner fence and lower hinge (adjacent), between lower outer fence and lower inner fence (out), less than lower outer fence (far out), between upper hinge and upper inner fence (adjacent), between upper inner fence and upper outer fence (out), and greater than upper outer fence (far out); an example of the alternative format is shown in Figure 5. Note that observations that fall under out and far out are considered as outliers.

## 4. Results

### 4.1. Scenario 1

Results from Scenario 1 are displayed in Figures 6 and 7 in the form a “numeric” tree diagram where infections involved more than 100 people. Out of 3580 infections, 38.66% of infections involved less than seven people, 14.25% of infections involved between 7 and 9 people, 22.96% of infections involved 9 to 17 people, 17.77% of infections involved 17 to 32 people, 4.66% of infections involved 32 to 47 people, and 1.7% of infections involved more than 47 people.

### 4.2. Scenario 2

Results from Scenario 2 are displayed in Figures 8 and 9 in the form of a “numeric” tree diagram where infections involved more than 60 people. Out of 8328 infections, 42.3% of infections involved less than three people, 12.55% of infections involved between 3 and 4 people, 20.58% of infections involved 4 to 7 people, 16.03% of infections involved 7 to 13 people, 5.4% of infections involved 13 to 19 people, and 3.13% of infections involved more than 19 people.

### 4.3. Scenario 3

Results from Scenario 3 are displayed in Figures 10 and 11 as a “numeric” tree diagram where infections involved more than five people. Out of 6742 infections, 71.49% of infections involved only one person, 21.61% of infections involved between 1 and 2 people, 5.12% of infections involved 2 to 3.5 people, 1.66% of infections involved 3.5 to 5 people, and 0.12% of infections involved more than 5 people.

## 5. Conclusion

In the previous section, we introduced models used by researchers, namely, a hybrid model (combining a health resource demand model with a disease transmission model), Bayesian model, SEIR model for predicting health service utilization and deaths, mixed-effect nonlinear regression, and mixture model to predict the number of confirmed cases and deaths or to predict when the curve will flatten. Apart from performing tasks similar to time series forecasting techniques (i.e., predicting the number of confirmed cases), system dynamics methodology focuses on the feedback behaviour of variables within the system's closed loop and deals with how the internal feedback loops within the structure of a system create behaviour. In this article, we modified and expanded system dynamics methodology beyond ordinary or normal usage when building the model called “COVID-19 confirmed cases,” from which were derived Scenarios 1, 2, and 3.

Scenario 1 is best described as the condition before the implementation of MCO in which approximately 80% of the population did not follow or practice social distancing, and on average, 996 people (out of 1000) became infected after 5 days of the observation period. The results showed that 38.66% of infections involved less than seven people, 37.21% of infections involved between 7 and 17 people, and 24.13% of infections involved more than 17 people, which includes 6.36% of infections which involved more than 32 people (they are considered as outliers). Due to the constraints of the size of the diagram, only one example of infections involving more than 100 people is given.

Scenario 2 is best described as the condition when CMCO was implemented or enforced (or before MCO was implemented or enforced), wherein approximately 50% of the population did not follow or practice social distancing. On average, 998 people (out of 1000) became infected after a 5-day observation period; results revealed that 42.3% of infections involved less than three people, 33.13% of infections involved between 3 and 7 people, and 24.56% of infections involved more than seven people, which included 8.53% of infections which involved more than 13 people (they are considered as outliers). Due to the constraints of the size of the diagram, only one example of infections involving more than 60 people is given.

Scenario 3's best-described condition was when MCO was implemented or enforced, where approximately 10% of the population did not follow or practice social distancing, and on average, 186 people (out of 1000) got infected after a 5-day observation period; further, results showed that 71.49% of infections involved 1 person, 26.73% of infections involved between 1 and 3.5 people, and 1.78% of infections involved more than 3.5 people, which include 0.12% of infections which involved more than five people (they are considered as outliers). Due to the constraints of the size of the diagram, only one example of infections involving eight people is given.

In conclusion, the scenarios show, apart from close to the real-world results, detrimental effects of ignoring social distancing guidelines (in terms of the decreasing number of people infected as compliance with social distancing norms increases).

Other (statistical) analysis of Scenarios 1, 2, and 3 can be found in Figures 12–14. Histogram of density estimation is used mainly for presentation and exploration of data. It is a nonparametric approach and can be defined as $\hat{f}\left(X\right)=1/nh$ (no of *X*_*i*_ in the same bin as *X*) where the bin refers to the interval [*x*_0_ + *mh*, *x*_0_ + (*m* + 1)*h*]  [13] (the said results were produced by “Explore Data Analysis,” a statistical program developed using Java programming language) (refer to Figures 12–14). These figures show they did not meet the requirement for further testing (i.e., fitting or not fitting the normal or bell-shaped distribution [14]; an example of a normal, bell-shaped distribution is shown in Figure 15).

The following are the steps for comparing real data with Scenarios 1, 2, and 3 (as mentioned earlier, real data containing clusters and patients are strictly confidential and the ones presented in this article are extracted from news or press release):

**Step 1 .**

Scenario 1, 2, and 3 results presented in this article are plotted together (i.e., combining Figures 12–14).

**Step 2 .**

Real data, *X*, fulfills the following: Scenario 1 condition, if $\hat{f}\left(X\right)$ is the highest at Scenario 1; Scenario 2 condition, if $\hat{f}\left(X\right)$ is the highest at Scenario 2; Scenario 3 condition, if $\hat{f}\left(X\right)$ is the highest at Scenario 3; Scenario 1 and 2 conditions, if $\hat{f}\left(X\right)$ is the highest at Scenarios 1 and 2; Scenario 1 and 3 conditions, if $\hat{f}\left(X\right)$ is the highest at Scenarios 1 and 3; Scenario 2 and 3 conditions, if $\hat{f}\left(X\right)$ is the highest at Scenarios 2 and 3; and Scenario 1, 2, and 3 conditions, if $\hat{f}\left(X\right)$ is the highest at Scenarios 1, 2, and 3 ($\hat{f}\left(X\right)$ refers to *f*(*t*(*k*)) in Figures 12–14).

The above steps were applied to patients [15, 16] where both fulfilled the Scenario 1 condition ([15] reports patient “zero,” a senior employee of a company, who attended public activities, events, and meetings after returning from Shanghai, China while [16] reports patient “zero,” a male restaurant owner, who broke home quarantine rules after returning from Sivaganga, India). Note that, “contact-tracing” exercise involves listing all contacts with patient “zero” and testing them for COVID-19.

We used Winter's Exponential Smoothing [17, 18] (the said results were produced by “Ritatwoanalytics3,” an expert system developed using Java programming language) method (a commonly used method, in which the “tracing” mechanism or feature is unavailable) to model Malaysia's COVID-19 confirmed cases [19] (represented by fit_wes_1 in Figure 16) where the downward trend can easily be changed or converted into an upward trend if we (i.e., businesses and population) fail to follow the SOP and do not practice social distancing (which are the measures for preventing the spread of the virus). Letting our guard down can lead our country into a second “wave” of infections, which would nullify our previous efforts with devastating results as shown in Scenarios 1 and 2.

Future research works can include the use of machine learning on the results given above.

## Figures and Tables

**Figure 1:** A (COVID-19 confirmed cases) model developed using system dynamics methodology.

**Figure 2:** Model “A” developed using the system dynamics methodology.

**Figure 3:** The results of Level_1 are displayed using a line plot.

**Figure 4:** Box plot properties.

**Figure 5:** Box plot is used to display statistical distribution, normal (0, 1), data. Note that normal (0, 1) data can be considered as equally distributed (only 0.3% are outliers).

**Figure 6:** Box plot showing Scenario 1 data.

**Figure 7:** Scenario 1 tree diagram showing the “level” of infections. Note that one of the branches in the tree diagram could represent patient “856” “family” members.

**Figure 8:** Box plot showing Scenario 2 data.

**Figure 9:** Scenario 2 tree diagram showing the “level” of infections.

**Figure 10:** Box plot showing Scenario 3 data.

**Figure 11:** Scenario 3 tree diagram showing the “level” of infections.

**Figure 12:** Scenario 1 density estimation. Three (skewed) peaks with differing densities are observed.

**Figure 13:** Scenario 2 density estimation. One (skewed) peak is observed.

**Figure 14:** Scenario 3 density estimation. Four skewed peaks with differing densities are observed.

**Figure 15:** Normal (0,1) density estimation.

**Figure 16:** Malaysia's confirmed COVID-19 cases (actual, represented by “Malaysia_confirmed,” and prediction, represented by “Fit_wes_1”).

## Data Availability

Real data is available in a public repository. Simulated data will be provided upon request.
